RETRACTED

# Pentoxifylline Can Reduce the Inflammation Caused by LPS after Inhibiting Autophagy in RAW264.7 Macrophage Cells

**DOI:** 10.1155/2021/6698366

**Published:** 2021-03-15

**Authors:** Danping Ruan, Sinan Deng, Zhonglong Liu, Jie He

**Affiliations:** ^1^Department of Stomatology, Minhang Branch, Zhongshan Hospital, Fudan University, Shanghai, China; ^2^Department of Oral and Maxillofacial-Head and Neck Surgery, Ninth People's Hospital, Shanghai Jiao Tong University School of Medicine, Shanghai Key Laboratory of Stomatology & Shanghai Research Institute of Stomatology, National Clinical Research Center of Stomatology, Shanghai, China

## Abstract

Pentoxifylline (PTX), as a methylxanthine derivative and nonspecific phosphodiesterase inhibitor, has the characteristics of anti-inflammatory and partial inflammatory process inhibition. However, the regulatory effect of PTX on inflammatory cytokines is unclear. Autophagy can regulate the activation of inflammasomes and then inhibit inflammation as previously described. Our study attempts to explore the relationship between autophagy and PTX-mediated regulation of inflammasome suppression. Macrophage-like RAW264.7 cells were studied as the *in vitro* macrophage model. We investigated the anti-inflammatory effect caused by PTX with time and dose response against the LPS-induced inflammatory factors (TNF-*α*, IL-1*β*). Western blot detected the levels of autophagy-related proteins Beclin-1 and LC3, as well as the signal pathways of AMPK and p-AMPK. Fluorescence microscope and transmission electron microscope were used to observe the autophagy bodies in cells influenced by PTX. The autophagy in cells inhibited by PTX exhibited dose- and time-dependent effects, and PTX alleviated LPS-induced inflammation caused by retarded autophagy. Furthermore, in RAW264.7 macrophage cells, our data indicated that AMPK signaling perhaps functioned importantly in repressed autophagy. In addition, in RAW264.7 macrophages, our data suggested that AMPK signaling might play an important role in inhibiting autophagy during the process of PTX ameliorating LPS-mediated inflammation.

## 1. Introduction

Inflammation is a complex pathological reaction, which resulted from multiple physical responses from the immune system when exposed to external injury or infection [1, 2]. Despite the fact that inflammation could compensate the wound, it was sometimes regarded as a protective process. In some cases, reduction of inflammation is of usefulness, but not usually essential. Macrophages originating from peripheral blood monocytes play fundamentally in cellular immunity and possess numerous complicated performances in specific and nonspecific inflammatory process, consisting of surveying objective organisms, chemotaxis, phagocytosis, and damage [3–6]. Multiple soluble factors, such as several secreted polypeptides (also known as macrophage-derived inflammatory cytokines), could lead to inflammation. Some of them, such as proinflammatory cytokines, could aggravate disease [7–9], while others, such as anti-inflammatory cytokines, were conducive to wound healing and also reduced inflammation [9–11]. Proinflammatory cytokine stimulated systemic inflammation, such as interleukin-1 (IL-1) and tumor necrosis factor alpha (TNF-*α*) [12, 13].

RETRACTED

Autophagy is a basic steady-state process through which cells decompose their assembly [14]. Recently, increasing evidences have suggested that autophagy displayed an important role in inflammation by affecting the development, homeostasis, and survival of inflammatory cells *in vivo* including macrophages, neutrophils, and lymphocytes, along with the transcription and secretion of many cytokines [15–17]. Monkkonen and Debnath found out that the pathways included in inflammation curbed or promoted autophagy in a context-dependent manner. Conversely, autophagy retarded or pushed inflammation in numerous carcinomas [18]. As Haq et al. demonstrated, identifying newly produced autophagy regulators in gut inflammation probably promoted new therapeutic regimes for intestinal inflammatory diseases [19]. Autophagy can raise or reduce disparate sections of identical inflammatory signaling concatenation in a context-dependent manner [20]. Autophagy is an extremely conservative homeostasis and inducible process that affects several aspects of the immune system, and is necessary for macrophages production and activation (comprising migration of monocyte/macrophage and differentiation of monocyte into macrophages), making autophagy become an appealing therapeutic target to further modulate macrophage response and a promising strategy for anticancer treatment [21]. AMP-activated protein kinase (AMPK) is a central mediator of cellular energy homeostasis, playing pivotal roles in regulating proliferation, metabolism reprogramming, autophagy, apoptosis, and cell differentiation. The kinase is activated in response to stresses that deplete ATP supplies such as low glucose, hypoxia, ischemia, and heat shock.

Pentoxifylline (PTX, C_13_H_18_N_4_O_3_), a methylxanthine derivative originally introduced for its rheologic effects, is a competitive nonselective phosphodiesterase inhibitor that can increase the decomposition rate of cyclic adenosine monophosphate (cAMP) and cyclic guanosine monophosphate (cGMP) and inhibit the synthesis of TNF and leukotriene. It is also an inhibitor with favorable anti-inflammatory effects and immunoregulatory properties [22, 23]. The drug can inhibit proinflammatory cytokine synthesis (IL-1, IL-6, IL-12, TNF-*α*) via lymphocytes and keratinocytes and retard the adhesion between leukocytes and endothelial cells or epithelial cells [24–26]. In humans, PTX demonstrated anti-inflammatory activity in some diseases such as cardiac surgery, acute radiation damage, chronic kidney disease, and HIV-infected patients [27–30]. Effects of pentoxifylline on inflammatory cytokine expression and inflammation-related disease inhibition were also found in animal models [31, 32]. PTX not only promotes the increase in anti-inflammatory cytokines towards a more stable immune phenotype but also prevents the production of proinflammatory cytokines [33, 34]. Therefore, it is a promising anti-inflammatory regulator candidate for ameliorating inflammatory environment. Sharma el al. indicated that activated ER stress response and autophagy were resistant to PTX-mediated apoptosis and thereby influenced the activity of PTX against cancer in human melanoma cells [35]. Nevertheless, there is little known towards the mediation role of PTX on inflammatory via regulation of autophagy, inflammasome, and the corresponding signaling pathways in macrophages.

RETRACTED

Given that autophagy participates in the process of inflammation and PTX displays anti-inflammatory activities though the inhibition of proinflammatory cytokines, the autophagy machinery that controls the influence of PTX against inflammatory needs to be further explored in a macrophage-like cell model. Our study tried to unearth PTX-induced regulation of the inflammatory responses and cytokine production by activating autophagy and inhibiting inflammasome as well as signaling pathway in RAW264.7 macrophage cells. We also hypothesized that the AMPK signaling played a crucial role in autophagy regulation and suppression of inflammation.

## 2. Materials and Methods

### 2.1. Reagents and Cell Culture

Pentoxifylline (PTX) was ordered from BD Biosciences (San Jose, CA, USA). *α*-MEM, FBS, penicillin, and streptomycin were ordered from Hyclone. 3-Methyadenine (3-MA) and LY294002 were ordered from Selleck Chemicals (Houston, TX, USA). Rabbit polyclonal anti-LC3, anti-IL-1-beta, anti-NLRP3, and anti-Beclin1 were obtained from Cell Signaling Technology Inc. (Danvers, MA, USA). Anti-TNF-*α*, anti-ERK1/2, and p-ERK1/2 were ordered from Abcam (Cambridge, MA, USA). Mouse polyclonal anti-GAPDH and rabbit polyclonal anti-P62 were ordered from Proteintech Group, Inc. Anti-*α*-tubulin rabbit polyclonal was ordered from Beyotime Biotechnology (Shanghai, China). Secondary antibodies were ordered from Thermo Scientific.

RETRACTED

Murine macrophage cells RAW264.7 were derived from the Institute of Biochemistry and Cell Biochemistry and Cell Biology (Shanghai, China). RAW264.7 were kept in DMEM containing 10% FBS and 5% penicillin/streptomycin at 37°C in a humidified 5% CO_2_ atmosphere.

### 2.2. Cell Viability Assay

1.0 × 10^3^ of cells in each well were inoculated in 96-well plates prior to PTX treatment. Cells were treated with 0, 0.2, 0.3, 0.5, and 0.8 mg/mL PTX at 24 h and 48 h. Then, the cell viability was determined with *α*-MEM containing Cell Counting Kit 8 (CCK-8) solution (Dojindo, Japan) in each well. The medium was then discarded and maintained for 2 h at 37°C in the dark. The absorbance value of 490 nm was detected by an ELISA reader.

### 2.3. PTX Time- and Dose–Response Detection

Whole-blood assays were conducted in many parts of this literature in order to reflect the aspect closest to physiological environment. Serum was not included. 0.5 mL of samples was maintained in 24-well plates with treatment of LPS (10 ng/mL) and PTX (20, 200, and 2,000 *μ*g/mL) for 4, 8, or 24 h at 37°C, 5% CO_2_. To detect cytokine production, supernatants were harvested, centrifuged, and maintained at -80°C until use at different postincubation time.

### 2.4. Cytokine Quantification in Supernatants

In the experiments, indicated cells pretreated with lipopolysaccharide (LPS) were then stimulated with 20 ng/mL interferon-*γ* (IFN-*γ*). The cells were exposed to 0, 50, 100, 200, and 400 ng/mL LPS in a concentration-dependent manner for 24 h; in addition, we also treated cells with 100 ng/mL LPS at 0, 3, 6, 12, and 24 h in a time-dependent manner. Through this two groups' analysis, we can determine the best treated concentration and time point. All samples were centrifuged after a specified time point of stimulation. Supernatants without cells were harvested and fast-frozen at −80°C until the following use. The IL-1*β* and TNF-*α* and other cytokine levels in supernatants were determined utilizing commercially available ELISA kits (Absin, Shanghai, China) as described in the manual. The threshold of detection sensitivity was 3.3 pg/mL for IL1-*β* and 3.7 pg/mL for TNF-*α*.

### 2.5. Western Blot Analysis

For per well, 1.0 × 10^6^ cells/mL were inoculated in Ø60 mm dishes as indicated. Whole cell lysate with 2% protease inhibitor and phosphatase inhibitors (Beyotime Biotechnology, China) was applied to harvest overall proteins. Bicinchoninic Acid (BCA) Protein Assay Reagent (Pierce, USA) was executed to determine protein concentrations. Approximately 20 *μ*g sample protein was loaded and ran on 10-15% SDS-PAGE gel, followed by transferring into polyvinylidene difluoride (PVDF) membrane (Millipore). 5% nonfat milk diluted in phosphate-buffered saline (PBS)/Tween 20 was used to block PVDF membrane for 1 h. PVDF membranes were rinsed three times with Tris-buffered saline Tween (TBST) and then incubated with primary antibody overnight at 4°C. At the following day, PVDF membrane was rinsed three times with TBST. Secondary antibodies were incubated with membrane for 1 h at ambient temperature.

RETRACTED

### 2.6. Immunofluorescence Staining and Fluorescence Microscope

The adenoviral constructs carrying mRFP-GFP-LC3 were obtained from HanBio Technology Co. Ltd. (Shanghai, China). Raw 264.7 cells were infected with adenovirus carrying mRFP-GFP-LC3 at MOI 200 upon cell confluence at approximately 80%. Macrophages were incubated in a 12-well plate with adenovirus diluted in 1 mL complete medium for 4 h in a37°C incubator as described by the manufacturers. The macrophages after transfection were incubated with DMEM containing 10% FBS overnight. Autophagosomes and autolysosomes in survival macrophages were counted by Cell Imaging Multi-Mode Reader (Cytation™5, BioTek Company, USA) with 40× image.

### 2.7. Transmission Electron Microscopy (TEM)

RAW264.7 cells were fixed with 2% glutaraldehyde for 2 h after 12 h PTX (0, 0.2, 0.5 mg/mL) treatment. After fixation, RAW264.7 incubated with 1% osmium tetroxide were dehydrated with gradient ethanol and then embedded in Epon-Araldite resin. The autophagosomes were visualized under the TEM (Tecnai G2 Spirit Bio TWIN, FEI Company, USA).

### 2.8. Statistical Analysis

The representative data was shown as the mean ± SEM of three separate experiments in triplicate one time. All data were processed and analyzed by *t*-test and ANOVA in SPSS 20 (Chicago, IL, USA). Obvious differences existing in different groups were shown as *P* < 0.05.

## 3. Results

### 3.1. Evaluation of Cell Viability after Pentoxifylline Treatment

The molecular structure of pentoxifylline (PTX) was shown in Figure 1(a). To get the safe concentrations (SCs) of PTX, we examined and evaluated the cytotoxicity of PTX with different concentrations (0, 0.2, 0.3, 0.5, and 0.8 mg/mL), as shown in Figure 1(b). After 24 h incubation, we found that cell survival had no significant difference among groups with PTX less than 0.5 mg/mL. Although with statistical significance between the 0.3 and 0.5 mg/mL groups, it holds no big difference with regard to the cell viability at a time point of 24 hours. Therefore, the concentration of PTX drug used in the following study was no more than 0.5 mg/mL.

### 3.2. LPS/IFN-*γ* Induced Inflammation in RAW264.7 Cells

LPS, a sort of endotoxin produced by outer membrane of bacteria, is famous as inducing inflammation [36], while interferon gamma (IFN-*γ*) is a pleiotropic molecule which can enhance proinflammatory signaling by activating macrophages for inflammatory cytokine level [37]. LPS stimulation of macrophages combined with IFN-*γ* can enhance macrophage activation and increase the expression of inflammatory factors [38, 39]. The lipopolysaccharide- (LPS-) primed inflammasome activation would induce some active proinflammatory cytokines and chemokine, such as interleukin-1*β* (IL-1*β*) and tumor necrosis factor *α* (TNF-*α*). Emerging data have shown that PTX can ameliorate inflammatory factor expression [40]. In order to set a model of IFN-*γ*/LPS-caused proinflammatory phenotype in RAW264.7 cells, IFN-*γ* (20 ng/mL) combined with 0, 50, 100, 200, and 400 ng/mL LPS were explored (Figures 2(a) and 2(c)). It was found that inflammatory factor (TNF-*α*, IL-1*β*) expression could be evidently raised when the LPS concentration was 100 ng/mL. When the concentration was increased to 200 ng/mL, the increasing effects of the expression of inflammatory factors were not obvious. Furthermore, we examined the influence of 100 ng/mL LPS and 20 ng/mL IFN-*γ* at different stimulating times (0, 3, 6, 12, and 24 h). Figures 2(b) and 2(d) showed that with the time gradient changes, significant inflammatory factor expression (TNF-*α*, IL-1*β*) was found at 24 h. Therefore, we chose the condition of IFN-*γ*/LPS-induced macrophage activation with LPS 100 ng/mL and IFN-*γ* 20 ng/mL, and the stimulation time was 24 h.

RETRACTED

### 3.3. PTX Ameliorated LPS-Caused Inflammatory Factors in RAW264.7 Cells

To verify that PTX has an inhibitory effect on LPS-mediated inflammation, we first pretreated macrophages with 0.2 and 0.5 mg/mL of PTX for 12 hours and then used 100 ng/mL+20 ng/mL of LPS/IFN-*γ* to treat cells for 24 hours. Inflammatory factor (IL-1*β* and TNF-*α*) level in the supernatant was measured by ELISA. Figures 3(a) and 3(b) illustrated that IL-1*β* and TNF-*α* level was inhibited with treatment of 0.2 and 0.5 mg/mL PTX, and the inhibited impact was significant when cells were treated with 0.5 mg/mL PTX. Then, PTX with a concentration of 0.5 mg/mL was adopted to pretreat cells with different times (6, 12, 24 hours) and followed by cotreating with LPS/IFN-*γ* for 24 h. With respect to the time of PTX treatment, the maximum inhibitory effect on the expression of IL-1*β* and TNF-*α* was found to be 12 h (Figure 3(c)). Furthermore, we maintained PTX treat time with 12 h, altered PTX with 0.2, 0.3, and 0.5 mg/mL, and then stimulated by LPS/IFN-*γ* for 24 h. It was found that as the PTX concentration increases, the inhibitory effect on IL-1*β* and TNF-*α* increases accordingly, and the inhibitory effect is significant after treatment of PTX of 0.5 mg/mL within the safe usage. The data indicated that 0.5 mg/mL PTX had significant inhibitory effect on LPS-mediated inflammation in RAW264.7 cells.

RETRACTED

### 3.4. PTX Inhibited Autophagy in RAW264.7 Cells in a Dose- and Time-Dependent Manner

Autophagy, being a regulation process of the innate immune system, is thought to modulate inflammatory cytokine generation [14–16]. Whether PTX had influence on the regulation of macrophage autophagy or not was checked in our following experiments. RAW264.7 cells were treated with 0.5 mg/mL PTX at 0, 6, 12, and 24 h. Autophagy-related protein (LC3, P62, and Beclin1) expressions were measured by Western blotting.  Figure 3(a) showed that with the increase of the treatment time, the expression of LC3 increased. Similarly, the expression of SQSTM1/P62 also increased accordingly. However, the expression of the autophagy-related protein Beclin1 decreased (Figure 3(b)). With respect to the cells treated with PTX of 0, 0.2, 0.3, and 0.5 mg/mL for 12 hours, LC3 and SQSTM1/P62 expression increased with raised drug concentration (Figure 3(c)), while Beclin1 expression was significantly reduced (Figure 3(d)). Therefore, we make a hypothesis that it might be the effects of PTX on macrophages that blocked the autophagy flux of the cells and thus suppressed the autophagy of the cells.

The LC3 proteins functioned critically in autophagy, and the localization of these proteins to autophagosomes can be used as a general marker for the accumulation of autophagosomes during inhibition of autophagic flux. To facilitate the high-throughput screening of autophagy-related PTX on macrophage cells, the RFP-GFP-LC3 construct was transfected into RAW264.7 cells. Then, GFP-RFP-LC3-transfected macrophages were treated with PTX of different concentrations (0, 0.2, and 0.5 mg/mL), and the autophagy flux situation image verifying RFP-GFP-LC3 expression in living cells was obtained with a fluorescent microscope (Figure 4(a)). When the concentration of PTX drug increased, the number of intracellular autophagosomes (yellow) was increased, and accordingly, the number of corresponding autophagolysosomes (red) was increased. Furthermore, the size and number of autophagic bodies were observed by electron microscopy [41].

It was found that with the concentration of PTX increasing, the number of intracellular autophagosomes (large arrows) increased, and so did the number of autophagolysosomes (small arrows). The experimental results of autophagy-related protein expressions, immunofluorescence tracking, and electron microscopy examinations all confirmed that the autophagy of RAW264.7 cells was blocked by PTX, which supports the hypothesis that PTX might block the autophagy flux of macrophage cells and thus result in the autophagy of the cells suppressed.

RETRACTED

### 3.5. PTX Ameliorated LPS-Induced Inflammation by Reducing Autophagy in RAW264.7 Cells

NLRP3 is a critical component of the inflammasome process [42]. There has been an increasing research concern on the crosstalk between autophagy and inflammation [20]. NLRP3 is found in autophagosomes upon activating inflammasome. To explore the feature of autophagy in determining the anti-inflammatory sensitivity of RAW264.7 cell response to PTX agent, we first examined the activity of autophagy in RAW264.7 cells with treatment of autophagy inhibitors like 3-methyladenine (3-MA, 5 mM) or LY294002 (5 *μ*M) with 0.5 mg/mL PTX and 100 ng/mL LPS. As shown in Figures 5(a) and 5(b), under the presence of 3-MA or LY294002, the stimulation with PTX obviously reduced IL-1*β* and TNF-*α* secretion to the supernatant of RAW264.7 cells in an intensity-dependent manner (^#^*P* < 0.05 or ^###^*P* < 0.001 compared to LPS+IFN-*γ*-treated cells). These results indicate that PTX might play its anti-inflammation role though autophagy regulation to a certain extent. In addition, NLRP3 is a critical component of the inflammatory process. After the pretreatment of LPS-treated RAW264.7 cells with autophagy inhibitors (3-MA or LY294002) or null, we found that 0.5 mg/mL PTX could decrease the proinflammatory cytokine (TNF-*α*) level and reduce NLRP3 level through autophagy inhibition. In summary, the results above imply that PTX influence on autophagy inhibition of RAW264.7 cells would present crucially in suppressing IL-1*β* and TNF-*α* secretion. The effects on IL-1*β* and TNF-*α* secretion were due to differences in inflammasome activation. To confirm this finding, we next used autophagy inhibitors to block AMP-activated protein kinase (AMPK) signaling to investigate to correlation of autophagy regulation and suppression of inflammation by PTX in RAW264.7 cells.

### 3.6. AMPK Signaling Pathway Displays Crucially in Regulating Autophagy and PTX Anti-Inflammation

Adenosine 5′-monophosphate–activated protein kinase (AMPK), a vital metabolic modulator of cellular and organismal process, impeded inflammation. Drug-induced activation of AMPK kinase could protect against inflammation [43, 44]. The cell autophagy can be coordinated by the AMPK signaling pathway [45]. To investigate the possible molecular mechanism of the relationship of PTX anti-inflammatory and autophagy, we explored the AMPK signaling pathway in autophagy and PTX anti-inflammatory in macrophages. The macrophage treated with PTX of 0.5 mg/mL was used as control.  Figure 6(a) showed that p-AMPK expression in cells treated with LPS+IFN-*γ* was obviously increased. However, p-AMPK expression was dramatically inhibited in cells pretreated with PTX.

RETRACTED

The results demonstrated that the AMPK signaling pathway of macrophages was suppressed by PTX. In accordance with the addition of the AMPK pathway activator A-769662, the expression of autophagy-related proteins LC-3 and Beclin1 was also increased (Figures 6(b) and 6(c)), which demonstrated the effect of AMPK signaling pathway involved with autophagy induction. In addition, the expression of TNF-*α* and NLRP3 in PTX pretreatment cells was dramatically lower relative to that in the LPS+IFN-*γ* group (Figure 6(d)), while with the addition of the AMPK pathway promoter A769662, the expression of TNF-*α* and NLRP3 increased obviously, and the anti-inflammatory effect of PTX was suppressed. The data indicated that the inhibition of PTX anti-inflammatory effects was related with the activated AMPK signaling pathway. Therefore, the AMPK pathway perhaps displayed an important role in the mechanism of PTX inhibiting autophagy and anti-inflammatory effect.

## 4. Discussion

PTX, approved by FDA, was applied in anti-inflammatory therapy. PTX can suppress proinflammatory cytokine gene transcription, such as TNF-*α*, but increase anti-inflammatory expression, such as IL-10 [25, 37], and it also inhibits other cytokines' key roles in inflammation such as IL-1*β* and IL-6 [31, 33]. However, it is still elusive whether PTX modulated the inflammatory responses via activating autophagy, inhibiting inflammasome, and the signaling pathway in macrophages. Our study illustrates that PTX inhibited autophagy in a dose- and time-dependent manner, and PTX ameliorated LPS-caused inflammation by reducing autophagy in RAW264.7 macrophage cells, and the AMPK signaling played a crucial role in autophagy regulation and PTX suppressed inflammation.

Inflammation is produced in the body upon exposure to injury or pathological infection. The adaptive immune system, particularly DCs and T cells, functioned primarily and specifically to regulate the inflammatory response. Macrophages are major participants in innate immune responses. The proinflammatory factors, such as cytokines and chemokines, are generated during infections or stimulus of inflammation. IL-1*β* and TNF-*α* are typical proinflammatory cytokines widely used in the study of inflammation-related diseases. Therefore, IL-1*β* and TNF-*α* were investigated to further confirm the success of LPS-primed inflammasomes activation in RAW264.7 macrophage cells (Figure 2). LPS-motivated IL-1*β* maturation in RAW264.7 cells was dramatically upregulated by 50 and 100 ng/mL of PTX at 3, 6, and 24 h as shown in Figures 2(a) and 2(b). Meanwhile, TNF-*α* activated by LPS-primed inflammasome in macrophages was significantly upregulated which was consistent with both dose (50, 100 ng/mL) and time (3, 6, 12, and 24 h), shown in Figures 2(c) and 2(d).

RETRACTED

As a nonspecific phosphodiesterase inhibitor, PTX would heighten intracellular cAMP and anti-inflammatory cytokine levels but reduce proinflammatory mediator production [22, 23]. In this study, our results indicated the maximum inhibited influences on IL-1*β* and TNF-*α* expression when treated with 0.5 mg/mL of PTX for 12 h (Figure 3). Similarly, Kalaiselvan [46] reported triphala (0.1–0.3 mg/mL) largely curbed inflammatory mediator production (e.g., TNF*α*, IL-1*β*) in a dose-related manner [38].

Cells could decompose their assembly by autophagy, which is a fundamental eukaryotic homeostatic process. NLRP3 is a key sensor molecule in the inflammasome activity [42]. Recently, current advances suggested that the pathway and proteins of autophagy exhibited a pivotal role in immunity and inflammation [20]. Many studies have confirmed that the effects of autophagy on inflammation have a two-way effect. On the one hand, autophagy might confront the inflammatory response by removing inflammatory protein aggregates and downregulating proinflammatory cytokines of tissue damage; on the other hand, autophagy would activate the inflammasome to produce a lot of inflammatory factors, thus accelerating the inflammation process. After balancing positive and negative sides of immunity and inflammation, autophagy could be regarded as a protector for infection, autoimmunity, and inflammation [14–17]. Our findings indicated that autophagy regulation probably contributed to therapeutic interventions towards diseases with inflammation. However, PTX performs the anti-inflammatory responses through autophagy activation as well as signaling pathways of inflammasome inhibition are still not well-known. Considering autophagy-related protein (LC3, P62, and Beclin1) expression, immunofluorescence tracking, and electron microscopy examinations (Figures 7 and 4), we found out that the PTX inhibited autophagy of RAW264.7 cells in a manner of dose and time dependence. Furthermore, when autophagy inhibitors 3-MA and LY294002 were added to PTX-treated cell, the PTX alleviated LPS-induced inflammation by reducing the proinflammatory cytokine (TNF-*α*, IL-1*β*) level. NLRP3 expression was greatly ablated (Figure 5). Therefore, PTX could block the autophagy flow of autophagic cells, and its inhibitory effect on LPS-mediated inflammation was significant in autophagy-inhibited cells.

RETRACTED

The AMPK signaling pathway functioned importantly in energy homeostasis and metabolism [44]. Some previous studies have shown that AMPK signaling perhaps functioned importantly in activated inflammatory body modulation. For example, Kim et al. [40] showed that adiponectin hindered LPS-caused activated inflammasomes in macrophages via inducing autophagy and activating the AMPK signaling pathway. Similarly, our data suggested that AMPK signaling displayed an important role in the regulation of PTX-mediated autophagy and inflammation (Figure 6). It is interesting that our data indicated that PTX inhibited the AMPK signaling pathway in macrophages, and it would cause anti-inflammatory response by inhibiting this pathway to suppress autophagy flow. Since the AMPK pathway links energy sensing to the anti-inflammatory signaling pathway, when autophagy was being inhibited, the formation of autophagosomes should be reduced. Similarly, Xie et al. reported that MAPK/ERK signaling pathways participated in the regulation of BRF1-mediated inhibition of LPS-induced inflammatory factor level and the autophagy flux in macrophage [47].

In summary, pentoxifylline suppresses inflammation in LPS-caused RAW264.7 macrophage cells that are relying on proper treatment time and dose. The autophagy in cells inhibited by PTX was found with dose and time dependence, and PTX alleviated LPS-induced inflammation which was caused by the downregulation of autophagy. Furthermore, AMPK signaling might display important function in autophagy inhibition during the process of PTX attenuating LPS-caused inflammation in RAW264.7 macrophage cells. New insight into the regulation basis of inflammation and autophagy will provide new perspective of anti-inflammatory drugs. Although the process of PTX inhibiting the AMPK signaling correlated with the number of autophagosomes followed by dose and time dependence in RAW264.7 cells, the phenomenon of AMPK inhibition and autophagosome increase might involve other pathways, which deserves further study in the future.

## Figures and Tables

**Figure 1:** (a) Molecular structure of pentoxifylline (PTX). (b) CCK8 assay detected RAW264.7 cell viability with 0, 0.2, 0.3, 0.5, and 0.8 mg/mL PTX treatment after 24 h and 48 h (^∗^*P* < 0.05 and ^∗∗^*P* < 0.01, compared to control).

**Figure 2:** LPS-caused inflammasome activation in macrophage under different conditions detected with enzyme-linked immunosorbent assay (ELISA) among supernatants. The IL-1*β* expression level was influenced by (a) a concentration-treatment manner (0, 50, 100, 200, and 400 ng/mL), and (b) a time-dependent manner (0, 3, 6, 12, and 24 h) treating with 100 ng/mL LPS and 20 ng/mL IFN-*γ*. The TNF-*α* expression level affected by (c) a concentration-treatment manner (0, 50, 100, 200, and 400 ng/mL) and (d) a time-dependent manner (0, 3, 6, 12, and 24 h) treating with 100 ng/mL LPS and 20 ng/mL IFN-*γ* (^∗∗∗^*P* < 0.001 compared to control, ns means no significance when compared to 100 ng/mL LPS-treated group).

RETRACTED

**Figure 3:** The content of IL-1*β* and TNF-*α* in supernatants was examined with ELISA. RAW264.7 cells were firstly treated with 0.2 mg/mL PTX (a) and 0.5 mg/mL (b) for 12 h, respectively, and then treated with 100 ng/mL LPS and 20 ng/mL IFN-*γ*. After 24 h incubation, carefully remove the medium without disturbing the layer of cells and collect the supernatant for ELISA analysis (^∗∗∗^*P* < 0.001; ^##^*P* < 0.01; ^###^*P* < 0.001). (c) The influences of pretreatment of PTX on the expression of IL-1*β* and TNF-*α* in RAW264.7 cells. The cells were firstly treated with 0.5 mg/mL of PTX for 6, 12, and 24 h, respectively. Then, cells were treated with 100 ng/mL LPS and 20 ng/mL IFN-*γ* for 24 h. After that, the cellular proteins were collected and examined by Western blotting. (d) The effects of PTX pretreatment concentration on protein expression of IL-1*β* and TNF-*α* in RAW264.7 cells. The cells were pretreated with 0.2, 0.3, and 0.5 mg/mL PTX for 12 h, respectively, and then treated with 100 ng/mL LPS and 20 ng/mL IFN-*γ* for 24 h. After that, the cellular proteins were collected and detected by Western blotting. Both in (c) and (d) the *α*-tubulin was the internal control, and quantitative analyses of protein expressions are represented by a bar graph (^∗∗∗^*P* < 0.001; ^###^*P* < 0.001).

**Figure 4:** Morphological observation of autophagy after PTX stimulation. (a) Fluorescence microscope observation of autophagy bodies (yellow) and autophagy lysosomes (red) affected by PTX concentration in cells and the GFP-RFP-LC3-transfected RAW264.7 cells treated with different PTX (0, 0.2, and 0.5 mg/mL). (b) Electron microscopy of autophagic bodies. RAW264.7 cells treated with different PTX (0, 0.2, and 0.5 mg/mL) were visualized by transmission electron microscopy. In control roots, few vesicles are apparent within the vacuole as they are immediately degraded. The autophagic bodies (big arrows) and autophagic lysosomes (small arrows) could be clearly observed.

**Figure 5:** (a) IL-1*β* and (b) TNF-*α* level in supernatants of RAW264.7 cells treated with PTX with or without autophagy inhibitor 3-MA/LY294002 was measured by ELISA. The cells were pretreated with 0.5 mg/mL PTX with or without autophagy inhibitor 3-MA and LY294002 for 12 h and then treated with 100 ng/mL LPS and 20 ng/mL IFN-*γ* for 12 h. Finally, the supernatants were collected for ELISA measurement (^∗∗∗^*P* < 0.001; ^#^*P* < 0.05, ^###^*P* < 0.001; ^$$^*P* < 0.01). (c) TNF-*α* and NLRP3 protein level in RAW264.7 cells cultured with or without the autophagy inhibitor 3-MA/LY294002 detected by Western blotting, and *β*-actin was the internal control. The cells were firstly treated with 0.5 mg/mL PTX for 12 h and then treated with 100 ng/mL LPS and 20 ng/mL IFN-*γ* for 12 h. The quantitative analysis of different protein expressions is shown by a bar graph (^∗∗^*P* < 0.01, ^∗∗∗^*P* < 0.001; ^#^*P* < 0.05, ^###^*P* < 0.001; ^$^*P* < 0.05, ^$$^*P* < 0.01).

**Figure 6:** (a) AMPK and p-AMPK protein level in RAW264.7 cells detected by Western blotting. The cells were initially treated with 0.5 mg/mL PTX for 12 h and then treated with 100 ng/mL LPS and 20 ng/mL IFN-*γ* for 6 h (^∗^*P* < 0.05; ^###^*P* < 0.001). (b, c) LC3 and Beclin 1 protein level in RAW264.7 cells cultured with or without the activator A-769662 of AMPK signaling pathways detected by Western blotting, and *β*-actin expression was the internal control. The cells were pretreated with PTX (0.5 mg/mL) for 12 h. The quantitative analysis of different protein expressions is shown by a bar graph (^∗^*P* < 0.05, ^#^*P* < 0.05, ^##^*P* < 0.01, ^###^*P* < 0.001). (d) TNF-*α* and NLRP3 protein level in RAW264.7 cells with or without activator A-769662 of AMPK signaling pathways was examined by Western blotting; and *β*-actin expression was the internal control. The cells were initially treated with 0.5 mg/mL PTX for 12 h and then treated with 100 ng/mL LPS and 20 ng/mL IFN-*γ* for 6 h. The quantitative analysis of different protein expressions is shown by a bar graph (^∗∗∗^*P* < 0.001; ^##^*P* < 0.01; ^##^*P* < 0.01, ^###^*P* < 0.001).

RETRACTED

**Figure 7:** Western blotting analysis of the effects of PTX (0.5 mg/mL) treatment time (0, 6, 12, and 24 h) on protein expression of (a) LC3 and SQSTM1/p62 and (b) Beclin1 and the concentration (0.2, 0.3, and 0.5 mg/mL) influence of PTX treatment for 12 h on protein expression of (c) LC3 and SQSTM1/p62 and (d) Beclin1 in RAW264.7 cells. *β*-Actin was the internal control (^∗^*P* < 0.05, ^∗∗^*P* < 0.01, and ^∗∗∗^*P* < 0.001 compared to control).

## Data Availability

The data that support the findings of this study are available with approval from the author.

## Supplementary Materials

Supplementary Materials PTX display an obvious inhibited influence on inflammatory factor expression caused by LPS-stimulated macrophages through autophagy suppression, in which the AMPK signaling pathway involved in the autophagy flux.
